# Bone Organic-Inorganic Phase Ratio Is a Fundamental Determinant of Bone Material Quality

**DOI:** 10.1155/2021/4928396

**Published:** 2021-10-31

**Authors:** Yunhua Luo, Ogheneriobororue Amromanoh

**Affiliations:** ^1^Department of Mechanical Engineering, University of Manitoba, Winnipeg, Canada; ^2^Department of Biomedical Engineering, University of Manitoba, Winnipeg, Canada

## Abstract

**Background:**

Bone mineral density is widely used by clinicians for screening osteoporosis and assessing bone strength. However, its effectiveness has been reported unsatisfactory. In this study, it is demonstrated that bone organic-inorganic phase ratio is a fundamental determinant of bone material quality measured by stiffness, strength, and toughness.

**Methods and Results:**

Two-hundred standard bone specimens were fabricated from bovine legs, with a specialized manufacturing method that was designed to reduce the effect of bone anisotropy. Bone mechanical properties of the specimens, including Young's modulus, yield stress, peak stress, and energy-to-failure, were measured by mechanical testing. Organic and inorganic mass contents of the specimens were then determined by bone ashing. Bone density and organic-inorganic phase ratio in the specimens were calculated. Statistical methods were applied to study relationships between the measured mechanical properties and the organic-inorganic phase ratios. Statistical characteristics of organic-inorganic phase ratios in the specimens with top material quality were investigated. Bone organic-inorganic phase ratio had strong Spearman correlation with bone material properties. Bone specimens that had the highest material quality had a very narrow scope of organic-inorganic phase ratio, which could be considered as the “optimal” ratio among the tested specimens.

**Conclusion:**

Bone organic-inorganic phase ratio is a fundamental determinant of bone material quality. There may exist an “optimal” ratio for the bone to achieve top material quality. Deviation from the “optimal” ratio is probably the fundamental cause of various bone diseases. This study suggests that bone organic-inorganic phase ratio should be considered in clinical assessment of fracture risk.

## 1. Introduction

Bone fracture is a common health concern among elderly people over the world, mainly due to the prevalence of osteoporosis and accident fall in the population [1–4]. Bone strength is a key mechanical property for the assessment of fracture risk. A direct and reliable way for the determination of bone strength is by mechanical testing, which is however invasive and not applicable to the human body. Bone density (BD) has been established as an indirect way to estimate bone strength. Extensive experimental studies have shown that at the material level, there is a relationship between bone strength and BD [5–8], and BD can be noninvasively measured by imaging technologies such as dual energy X-ray absorptiometry and quantitative computed tomography [9–11]. Bone mineral density is recommended by the World Health Organization as a gold reference for the screening of osteoporosis and for the assessment of fracture risk [12, 13]. It is important to note that bone mineral density refers to the content of inorganic minerals in a unit bone volume, while BD includes all the material compositions.

Numerous clinical studies have shown that bone mineral density is not a reliable predictor of fracture risk [14–19]. Bone fractures often occur in people who are not in high risk if assessed by bone mineral density. With a close examination of a variety of methods developed for the prediction of fracture risk, de Bakker et al. [20] pointed out the importance of bone material properties in determining whole-bone mechanics. Based on a critical analysis of the biomechanical variables involved in clinical assessment of hip fracture risk, it was identified that the oversimplified relationship between bone strength and bone material compositions probably has substantial adverse effect on the accuracy of the biomechanical models [21]. Bone compositions play different roles in regulation of bone strength and other mechanical properties [22, 23]. The inorganic minerals mainly regulate bone stiffness and compressive strength, while the organic proteins primarily govern bone flexibility and toughness [24–26]. The existing bone elasticity-density relations have a sole density variable, which is not able to describe the composition difference in bones, and thus have numerous fundamental limitations. For example, the relations are found anatomic site-dependent [27]; they can not explain why old bones are more brittle than young bones even they have similar density [28], and why bones have different compressive and tensile strength [29, 30].

Our previous study has shown that bone material quality is dependent on the quality and quantity of organic and inorganic phases [31]. In this paper, it is further demonstrated that bone organic-inorganic phase ratio is a fundamental determinant of bone material quality measured by stiffness, strength, and toughness.

## 2. Materials and Methods

### 2.1. Consideration of Bone as an Organic-Inorganic Composite Material

Bone has complicated chemical and material compositions at the microscopic scale [32]. At the material level, bone is composed of inorganic minerals, organic proteins, and water [24]. About 90% of the minerals are hydroxyapatite, and 90% of the proteins are type I collagen protein [33, 34]. The proteins and water are combined in one phase but still collectively call them “organic” phase. Water exists in two forms in bone, i.e., water bonded with proteins and free water in pores [35]. It is difficult to separate bounded and free water in bone; the concern is that excessive removal of bounded water can degrade proteins and thus substantially change their mechanical properties [35, 36]. By considering bone as an organic-inorganic composite material, the organic and inorganic content can be determined by ashing. Organic matters including water are burned out during ashing, while inorganic minerals remain.

### 2.2. Bone Specimens

Forty bovine leg bones (10 healthy cows, age of 12 to 18 months) were acquired from local certified slaughterhouses. The harvested bones were immediately wrapped in air-tight plastic bags and stored in a freezer with the temperature set at -20°C. A specially designed method as described in Figure 1 was used to fabricate bone specimens. The bone specimens manufactured with this method are approximately along the femur axis, and the effect of bone anisotropy on mechanical properties is thus reduced. Two-hundred cylindrical specimens were manufactured. Experimental data were successfully measured from 173 specimens (length 28.5 ± 2.2 mm, diameter 7.8 ± 0.4 mm), including 95 cortical and 78 cancellous bones.

### 2.3. Mechanical Testing and Bone Ashing

Prior to mechanical testing, specimens were taken out from the freezer and dwelled in room temperature and humidity for four hours, so that bone temperature and moisture did not change anymore. The procedure that was applied to generate experimental data in this study is described as follows. Specimen length, diameter, and weight were measured using caliper and digital weight scale. Specimens were compressed until failure using an MTS Insight Electromechanical Testing System, see Figure 2(a), with a loading rate of 1.5 mm/minute. The testing system was periodically calibrated by a certified technician. Bone mechanical properties, including Young's modulus, yield stress, peak stress, and energy-to-failure, were automatically measured by the testing system. After mechanical testing, specimens were ashed in a muffle furnace (Fisher Scientific, Canada) under 700°C for 20 hours, compare Figure 2(b). Each specimen was ashed in a separate crucible with cover. The weight lost during the ashing was taken as the organic mass; the ash weight was measured and taken as the inorganic mass.

### 2.4. Statistical Analyses

To study the effect of organic-inorganic phase ratio on bone material properties, Spearman correlation and *p* value were calculated; nonlinear model fitting was conducted. A number of nonlinear models, including polynomials of different orders and exponential functions, were attempted to find out the best fitting.

To investigate statistical characteristics of organic-inorganic phase ratio in specimens of high material quality, specimen groups that had the top 10%, 20%, and 30% of density, Young's modulus, yield stress, peak stress, and energy-to-failure were identified; mean values and standard deviations of the ratios in the groups were calculated.

## 3. Results

Spearman correlation (*ρ*) and *p* value that show the correlations of BD, Young's modulus, yield stress, compressive strength, and energy-to-failure with organic-inorganic phase ratio are listed in Table 1.

Relationships between bone material properties and organic-inorganic phase ratio were found highly nonlinear. The models that had the best fitting with the experimental data were in the form of exponential function

(1) $$\begin{array}{c} y=a\cdot r^{b}, \end{array}$$

where *r* is the organic-inorganic phase ratio, *y* is one of the material properties shown in Table 1, and *a* and *b* are coefficients determined by nonlinear model fitting. The coefficients of determination (*R*^2^) were 0.85 for density, 0.85 for Young's modulus, 0.82 for yield stress, 0.88 for peak stress, and 0.70 for energy-to-failure. The nonlinear models together with the experimental data are shown in Figure 3.

Statistical characteristics of organic-inorganic phase ratios in the specimen groups of top 10%, 20%, and 30% of density, Young's modulus, yield stress, peak stress, and energy-to-failure are listed in Table 2.

The results show that bone organic-inorganic phase ratio had significant effect on the material properties (Table 1), and the effect was nonlinear (Figure 3), suggesting that a small deviation of the ratio from the means in Table 2 may substantially reduce bone material quality.

## 4. Discussion

Spearman correlations and *p* values in Table 1 show that bone organic-inorganic phase ratio has strong (*ρ*=-0.83 – -0.92) and significant (*p* < 0.001) correlations with bone material properties, suggesting that bone organic-inorganic phase ratio is an important determinant of bone material quality. By integrating the above finding with those from previous studies [8], one can produce a more complete picture (see Figure 4) regarding the dependence of bone material quality on bone composition. Several studies, which have been comprehensively reviewed by Helgason et al. [8], have evaluated the relationship between bone stiffness/strength and BD. This study further revealed that BD is dependent on organic-inorganic phase ratio, see Table 1 and Figure 3(a). Therefore, bone organic-inorganic phase ratio is a more fundamental determinant than BD in regulation of bone material quality. Correlations in Table 1 also show that, with the increasing of organic content, bone stiffness and strength would decrease, which is consistent with the mechanics of composite materials [37]. If the bone is considered as a two-phase composite, bone organic phase plays the role of the matrix, while the inorganic phase acts as the reinforcement or inclusion. The organic phase of bone, which mainly consists of type I collagen proteins, has much lower density, stiffness, and strength than the inorganic phase that is dominated by hydroxyapatite [38, 39]. Based on the mechanics of composite materials, a higher organic content would definitely result in lower stiffness and strength [37].

Results in Figure 3 and Table 2 further suggest that there exists a certain organic-inorganic phase ratio for bone to achieve top material quality. It is interesting to note that, if testing error is considered, the top material properties of the tested specimens were achieved by almost the same organic-inorganic phase ratio (see Table 2). For example, the ratio was between 0.61 and 0.62 for top 10% material properties, which can be considered as the optimal ratio in the tested specimens. The existence of optimal phase ratio is probably the result of balancing between the different roles of organic and inorganic phases in the regulation of bone material properties. First, collagen protein in extracellular matrix is the “house” for the accommodation of inorganic minerals, and a unit volume of collagen protein can only accommodate a certain amount of inorganic minerals [40]. Therefore, the quantity and quality of collagen protein determine the quantity of inorganic minerals that can be deposited in a bone. Either inadequate or excessive amount of collagen protein would result in a weak bone. Second, bone toughness is a more crucial property than bone strength to resist fracture [41] but has not been considered in the clinical assessment of fracture risk. In material science, toughness is the ability of a material to absorb mechanical energy and sustain deformation without fracturing. Material toughness is measured by the area under the stress-strain curve. In order to be tough, a material must be both strong and ductile, which are, respectively, governed by the bone inorganic and organic phases.

One limitation of this study is that only young and healthy bones were tested, due to the difficulty in the acquisition of diseased bovine bones. However, on the basis of composite material theory, it can be inferred that a higher organic-inorganic phase would improve bone ductility but compromise strength. On the other hand, a lower ratio would increase bone strength but also promote fragility. Emerging research evidence shows that imbalance between organic and inorganic phase is a fundamental cause of various bone diseases [24]. For example, osteomalacia, also referred as softened bone disease, is characterized by a low mineralization of bone matrix [42–44], or equivalently, the organic-inorganic phase ratio is abnormally high. In contrast, osteogenesis imperfecta, or brittle bone disease, is attributed to the deficiency of producing collagen protein in the body [45–47]; the bone thus has an abnormally low organic-inorganic phase ratio. Osteoporosis is a bone disease closely related to aging. With aging, the body has a reduced ability to produce new collagen proteins in remodeling [48–50], resulting in organic-inorganic phase ratio shifted to the lower side.

The findings from this study indicate that, to improve the clinical assessment of bone strength and fracture risk, it is necessary to measure bone protein content in addition to bone mineral density, which requires a noninvasive technique such as bone imaging. Existing bone imaging modalities such as magnetic resonance imaging and quantitative computed tomography can only measure either the organic or the inorganic content [11] but not both. Recent advances in water- and fat-suppressed projection imaging [51, 52] make it possible to noninvasively detect both organic and inorganic content, thus providing a feasible way for the implementation of the findings to clinical applications.

## 5. Conclusions

Based on the results in this study, it can be concluded that bone organic-inorganic phase ratio is a fundamental determinant of bone material quality, and there exists an “optimal” ratio for the bone to achieve top material quality. Deviation from the “optimal” ratio is probably the fundamental cause of various bone diseases. This study suggests that bone organic-inorganic phase ratio should be considered as a risk factor in clinical assessment of fracture risk.

## Figures and Tables

**Figure 1:** (a) Soft tissues were completely removed, and the bone was positioned in mold. (b) Mixed plaster of Paris was poured in. (c) After plaster consolidation, mold was removed. (d) The molded femur was transversely sliced in 30 mm thickness using a laser-guided mitre saw; bone specimens were cored from the slices using diamond coring bit of 8 mm diameter. (e) Information of each specimen, including animal, femur, anatomic site, and bone type, was recorded; the specimens were then labeled, wrapped with kitchen film, put in air-tight plastic container, and then stored in the freezer (-20°) before testing.

**Figure 2:** (a) Compression testing. (b) Bone ashing.

**Figure 3:** Variations of bone material properties with organic-inorganic phase ratio: (a) density; (b) Young's modulus; (c) yield stress; (d) peak stress; (e) energy-to-failure.

**Figure 4:** The dependence of bone material quality on organic-inorganic phase ratio.

**Table 1:** Spearman correlation (*p* value) between organic-inorganic phase ratio and bone material properties.

Material property	Spearman correlation *ρ* (*p* value)
Density	-0.89 (*p* < 0.001)
Young's modulus	-0.83 (*p* < 0.001)
Yield stress	-0.89 (*p* < 0.001)
Peak stress	-0.92 (*p* < 0.001)
Energy-to-failure	-0.85 (*p* < 0.001)

**Table 2:** Statistical characteristics of organic-inorganic phase ratio in groups of specimens having top material quality.

Material property	Top 10%		Top 20%		Top 30%	
	Mean (SD)	Range	Mean (SD)	Range	Mean (SD)	Range
Density	0.61 (0.03)	(0.54, 0.68)	0.62 (0.04)	(0.54, 0.77)	0.64 (0.06)	(0.54, 0.83)
Young's modulus	0.61 (0.01)	(0.54, 0.68)	0.62 (0.04)	(0.54, 0.72)	0.65 (0.07)	(0.54, 0.88)
Yield stress	0.62 (0.02)	(0.54, 0.71)	0.63 (0.05)	(0.54, 0.78)	0.65 (0.07)	(0.54, 0.88)
Peak stress	0.62 (0.04)	(0.54, 0.71)	0.62 (0.04)	(0.54, 0.72)	0.64 (0.06)	(0.54, 0.83)
Energy-to-failure	0.62 (0.05)	(0.54, 0.72)	0.63 (0.07)	(0.54, 0.79)	0.65 (0.12)	(0.54, 0.89)

## Data Availability

The experimental datasets produced by the current study are available from the corresponding author on reasonable request.
